The article "The Effects of Virtual Reality Training on Function in Chronic Stroke Patients: A Systematic Review and Meta-Analysis" was published in 2019. Journal: Biomed Res Int.

# The Effects of Virtual Reality Training on Function in Chronic Stroke Patients: A Systematic Review and Meta-Analysis

**DOI:** 10.1155/2019/7595639

**Published:** 2019-06-18

**Authors:** Han Suk Lee, Yoo Junk Park, Sun Wook Park

**Affiliations:** ^1^Department of Physical Therapy, Faculty of Health Science, Eulji University, 553 Sanseongdae Ro, Sujeong-gu, Seongnam, Gyeonggi-do 13135, Republic of Korea; ^2^Department of Physical Therapy, Samsung Seoul Hospital, 81 Irwon Ro, Gangnam-gu, Seoul 06351, Republic of Korea

## Abstract

**Objective:**

The aim of this study was to perform a meta-analysis to examine whether virtual reality (VR) training is effective for lower limb function as well as upper limb and overall function in chronic stroke patients.

**Methods:**

Three databases, OVID, PubMed, and EMBASE, were used to collect articles. The search terms used were “cerebrovascular accident (CVA),” “stroke”, and “virtual reality”. Consequently, twenty-one studies were selected in the second screening of meta-analyses. The PEDro scale was used to assess the quality of the selected studies.

**Results:**

The total effect size for VR rehabilitation programs was 0.440. The effect size for upper limb function was 0.431, for lower limb function it was 0.424, and for overall function it was 0.545. The effects of VR programs on specific outcomes were most effective for improving muscle tension, followed by muscle strength, activities of daily living (ADL), joint range of motion, gait, balance, and kinematics.

**Conclusion:**

The VR training was effective in improving the function in chronic stroke patients, corresponding to a moderate effect size. Moreover, VR training showed a similar effect for improving lower limb function as it did for upper limb function.

## 1. Introduction

Stroke is a major cause of death in the modern world; it also causes sensory, motor, cognitive, and visual impairments and restricts performance of activities of daily living (ADL) [1]. Motor impairments are observed in 80% of stroke patients, and these can include loss of balance and gait [2]. These problems are important targets of rehabilitation, because they reduce the ability of individuals to perform ADL and this result in impaired community activities [3, 4].

Most studies on balance and gait rehabilitation have shown positive effects. However, training-based methods often become tiresome are resource-intensive and require specialized facilities or equipment. Therefore, there is a demand for economical and safe methods of rehabilitation [2].

Virtual reality (VR) is defined by “the use of interactive simulations created with computer hardware and software to present users with opportunities to engage in environments that appear and feel similar to real world objects and events.” Participants interact with projected images, maneuver virtual objects and perform activities programmed into the task, giving the user a sense of immersion in the simulated environment. Various forms of feedback are provided through the environment, the most common being visual and auditory, to enhance enjoyment and motor learning through real-time feedback and immediate results [5]. VR training using these features has recently been widely used in the field of stroke rehabilitation [3]. VR training aims to improve neural plasticity by providing a safe and enriched environment to perform functional task-specific activities with increased repetitions, intensity of practice, and motivation to comply with the intervention [1].

In the field of stroke rehabilitation, VR training is reported to be mostly effective at increasing upper limb joint range of motion, improving sensation, muscle strengthening, reducing pain, and improving functional processes. Recently, various VR programs have been developed and implemented for the lower limbs as well as the upper limbs, and their effects are being tested. VR training for stroke patients has been shown to be safe and cost-effective at improving lower limb function, specifically improving balance, stair climbing speed, ankle muscle strength, range of motion, and gait speed [1]. Compared with existing treatment methods, it may be more effective at improving dynamic balance control and preventing falls in subacute and chronic stroke patients [6].

Treatment methods using VR provide a virtual environment for ADLs that are difficult to perform in a hospital, and therefore, it could be very effective at improving both upper limb and lower limb function. However, because the lower limbs have to support the weight of the body, various elements are required, including muscle strength and balance to control body weight, joint movements, and cognitive ability to integrate these other elements. Although studies related to VR training have been increasing in recent years, VR intervention has been used more extensively to improve upper limb function, which is relatively easier to apply than lower limb function.

Furthermore, doubts could be raised as to whether VR treatment methods for the lower limbs can improve these elements; these doubts related to lack of VR equipment or programs, as well as safety issues or dizziness during treatment. For this reason, we aimed to perform a meta-analysis as a scientific method to test the effects of uncertain treatment methods using statistical methods, in order to examine whether VR training is effective for lower limb function as well as upper limb function.

## 2. Methods

### 2.1. Study Search Procedures and Inclusion Criteria

Using the PICOS (Patients, Intervention, Comparison, Outcomes, Study designs) method [7], we investigated patients (P) who had been diagnosed with chronic stroke (more than 6 months after stroke); the intervention (I) was VR rehabilitation therapy, and we compared (C) this with a control group not receiving VR rehabilitation. The outcomes (O) were changes in upper limb function, lower limb function and overall function on daily activity as a primary outcome. Upper limb function was assessed if the chosen instrument measured the impact of upper limb function of individual as FMA-UL, muscle strength related to upper limb, JHFT (Jebsen Taylor Hand Function Test), Pinch ability related to hand, Wolf Motor Function Test, ROM related to upper limb, Kinematic data related to upper limb, Grooved Pegboard Test. MAS of upper limb, Motor Activity Log-quality of movement. Lower limb function was assessed if the chosen instrument measured the impact of lower limb function individual as gait variable like speed and cadence, the tools related to balance, Tinetti Performance Oriented Mobility Assessment, FMA-LL, MAS of lower limb, muscle strength test related to lower limb. Overall function was assessed if the chosen instrument measured the impact of total function of individual on every life style like functional independence measure, total FMA, Barthel index score, quality of life. Study design (S) was randomized control designs. Using OVID, PubMed, and EMBASE, during the same period, two researchers independently searched studies published in English from January 2000 up to June 2018. The search terms used were ‘cerebrovascular accident (CVA),' “stroke”, and “virtual reality” (Table 1), and discrepancies in the search results were resolved by consensus after a discussion.

A total of 1667 studies were retrieved from the databases after the first search. The inclusion criteria were as follows: studies of patients diagnosed with chronic stroke, studies using VR as a therapeutic intervention, studies that measured function-related changes, and studies that used a randomized controlled trial (RCT) design [8, 9]. The exclusion criteria were graduation theses, books, conference proceedings, single case studies, and quasi-randomized or other qualitative studies. Eventually, 21 articles were included in the meta-analysis based on the PRISMA protocol (Figure 1).

### 2.2. Quality Assessment

The PEDro scale [31] was used to assess the quality of the selected studies. PEDro scale scores of 9–10 are considered to be of excellent quality, scores of 6–8 points and 4–5 points to be of good and fair quality, respectively, and scores below 4 are of poor quality [32]. The mean PEDro scale score of the selected studies was 6.28 (range from 6 to 8), indicating good quality (Table 2).

### 2.3. Coding and Data Analysis

For data coding, the authors' names, year of publication, type of publication, research model, study participants, assessment instruments, type of program, and effects of the program were recorded by consensus between a physiotherapist and a meta-analysis expert. Data analysis was performed using CMA 2.0 (Biostat, Englewood, NJ, USA). Heterogeneity was assessed by means of the value of the I^2^ statistic, where an I^2^ value greater than 50% indicated significant heterogeneity. When there was little heterogeneity, pooled analyses were conducted using a fixed effects model. Likewise, when there was great heterogeneity between studies, a random effects model was used [33]. Data were synthesized using a meta-analytic method based on a random effects model due to the small studies even though the results of heterogeneity testing for the studies were not significant (Q(20) = 27.499, I^2^=27.269, p > 0.05) [7]. All effect sizes were changed to the Hedges g statistic because it contains a small sample bias correction [34, 35]. Sensitivity analysis is an analytical method that examines how results change according to the criteria and contents of analysis. We drop the study that score below 4 point in methodological quality of trials from the meta-analysis to confirm its effect on results for sensitivity analysis [7].

## 3. Results

### 3.1. Data and General Characteristics of the Selected Studies

We used 33 effect sizes from 21 studies. There were 562 patients in total. General information about the studies included in the analysis is shown in Table 3.

### 3.2. Testing for Publication Bias

In the analysis of publication bias, the funnel plot (Figure 2) was symmetrical, and a trim and fill analysis gave a result of 0.440 for both the observed and the adjusted values, 0.440 (0.360–0.520). When we tested Kendall's tau based on the method by Begg and Mazumdar (1994) [36, 37], there was no significant correlation (*τ* = .281, p > 0.05). Therefore, we were able to conclude that the studies in this analysis did not show publication bias.

### 3.3. Analysis of the Total Effect

To analyze the effects of VR rehabilitation programs, we calculated the effect size as the ‘standardized mean difference;' the total effect size for a random effects model was 0.440, corresponding to a moderate effect size [33], and this was statistically significant (p < 0.05) (95% CI: 0.360–520). A forest plot for all 21 studies is shown in Figure 3. Sensitivity analysis showed that the total effect size of the random effects model was 0.446 and the 95% confidence interval was 0.361-530, which was statistically significant. As a result of the sensitivity analysis, there is little difference in total effect size except for low quality research.

### 3.4. The Effects of VR Rehabilitation Programs on Functional Improvement

The effect size for upper limb function was 0.431, for lower limb function it was 0.424, and for overall function it was 0.545; these results were statistically significant (p≤0.001) (Table 4). Sensitivity analysis showed that the effect size of the upper limb function was the same as that of the overall function, and the effect size of the lower limb function was 0.432 (CI; 0.339-0.526), which was statistically significant. In other words, there was no significant difference in results except for low quality studies.

### 3.5. The Effects of VR Rehabilitation Programs on Specific Aspects of Functional Improvement

We compared the effects of VR programs on specific outcomes, and found that, in descending order, it was most effective for improving muscle tension, followed by muscle strength, ADL, joint range of motion, gait, balance, and kinematics. In particular, very large effect sizes were observed for improvements in muscle tension, muscle strength, and ADL. Statistically significant results were observed for all items (p < 0.05) (Table 5).

Sensitivity analysis showed the same results except for balance and gait, but there was no significant difference in balance and gait. In the case of the balance, the effect size of before and after sensitivity analysis were 0.364 (CI: 0.244-0.484) and 0.354 (CI: 0.226-0.482) respectively. In the case of gait, the effect size was 0.445 (CI: 0.309-0.582) before the sensitivity analysis, but the effect size was 0.469 (CI: 0.325-0.613) after the sensitivity analysis.

### 3.6. Analysis by Program Mode

In a meta-regression analysis by duration of intervention, the slope coefficient was 0.019 (95% CI: −0.022–0.061), and longer duration was associated with larger effect size; however, the slope coefficient was not statistically significant (P > 0.05). Nevertheless, the slope showed a high effect size as the duration approached 8 weeks (Figure 4). In a meta-regression analysis by weekly frequency of intervention, the slope coefficient was –0.016 (95% CI: −0.078–0.046), and as the frequency increased, the effect size decreased; h the slope coefficient was not statistically significant (P > 0.05) (Figure 5).

The sensitivity of the meta-regression analysis was 0.029 for the treatment duration and -0.012 for the frequency per week, which was not statistically significant.

## 4. Discussion

VR treatment methods are economical, provide clear motivation, can improve the effects of treatment, and can provide opportunities for the user to participate in a realistic environment resembling real objects and events by integrating multiple sensory stimuli through visual, auditory, tactile, and somatosensory systems [1, 3, 5, 14, 38]. For these reasons, VR rehabilitation training has recently emerged as an important method to promote functional recovery after a stroke.

We performed a systematic review and meta-analysis to investigate whether VR rehabilitation training is effective at improving function in chronic stroke patients, and observed moderate effect size (ES = 0.440). Aminov et al. [39] reported that VR provides additional benefits compared to conventional methods, and that it can bring immediate and long-term improvement in post-stroke motor function. We also observed moderate effect size for VR rehabilitation training, suggesting that this technique may be used as a complementary treatment method alongside traditional rehabilitation therapy.

When we performed a subgroup analysis of the effects on functional improvement, the effect size was moderate for upper limb function (ES = 0.431), lower limb function (ES = 0.424), and overall function (ES = 0.545). Therefore, VR rehabilitation training improved lower limb function, including balance and gait, to a similar degree as upper limb function in chronic stroke patients, and it also improved overall physical function. Previous studies reported that use of VR in chronic stroke patients produced significant improvements in functional balance, gait velocity, cadence, and stride length [1], and that performing VR training alongside balance and gait treatment was more effective for improving gait speed and TUG than balance and gait training alone [2]. Other meta-analyses suggested that VR training improves BBS and TUG in chronic stroke patients compared to conventional rehabilitation [3, 40]. Chen et al. [6] provided moderate evidence to support the claim that VR training is effective as a complementary therapy to a standard rehabilitation program to improve balance in chronic stroke patients; however the effects were unclear in acute or subacute stroke patients. In a systematic review, Moreira et al. [4] claimed that training using VR had potential as a method to improve gait parameters in chronic stroke patients, irrespective of the number of participants in the study, participant characteristics, and protocol diversity. Similarly, we found that, although VR programs can cause some discomfort, including dizziness [41], they are as effective at improving lower limb function as they are at improving upper limb function. This is thought to be because most programs included in the analysis consisted of game-based tasks, using equipment such as the Nintendo Wii or Xbox Kinect, meaning that subjects had little difficulty using the programs. Programs in the form of games have similar beneficial effects on upper limb function, lower limb function, and overall function.

Laver et al. [42] reported that VR and interactive video games were no better at improving upper limb function in stroke patients than was conventional treatment, and that their effects on gait speed, balance, participation, and quality of life were also unclear. Nevertheless, implementing VR training together with conventional treatment significantly improved upper limb function and helped improve ADLs in a similar way to extending the overall treatment duration. Most of the studies in our analysis also increased the overall treatment time by adding VR training to conventional treatment, and it is possible that this is the reason we observed effects for both the upper and lower limbs, despite most studies also using game-based programs.

When we investigated the effects of VR rehabilitation training on specific aspects of function in chronic stroke patients, we observed relatively strong effects on muscle tension (ES = 0.755) and muscle strength (ES = 0.722), but only moderate to relatively weak effects on (in descending order of effect size) ADLs, joint range of motion, gait, function, balance, and kinematics (ES = 0.627–0.274). Lee [43] reported that voluntary mobility training using Xbox Kinect improved muscle strength, resulting in improved ability to perform ADLs. In a meta-analysis by Laver et al. [42], VR was found to have a moderate size effect at improving ADLs. Meanwhile, in another systematic report and meta-analysis, Aminov et al. [39] reported that VR training had significant effects on body structure/function and activity level as a complementary measure to conventional treatment methods for post-stroke rehabilitation.

Like previous studies, we also found that VR training could be very helpful for improving muscle strength and ADL. This is thought to be because VR training can enhance high-intensity, repeated, task-oriented training typically used as an evidence-based intervention method in chronic stroke patients.

When we analyzed the effects of VR training by treatment duration, a longer duration was associated with a stronger effect, and analysis of the slope showed that a duration closer to 8 weeks resulted in a strong effect. However, it was not statistically significant (p=0.364).

Also, in the meta-regression analysis by weekly treatment frequency, a higher frequency was actually associated with a reduced effect. However, it was not statistically significant (p=0.614).

Given that physical adaptation to exercise usually occurs after 6–8 weeks [44], our results suggest that duration of at least 8 weeks is required to obtain an effect from VR. However, most of the studies included in our analysis had a duration of 6 weeks or less, and there were only three studies with a duration over 6 weeks. We believe that this is because the characteristics of chronic stroke patients make long-term VR treatment difficult. Nevertheless, researchers should consider the fact that a duration of at least 8 weeks is required for physical adaptation. In other words, it seems that there was not a significant difference in treatment effect because it took some time to adapt to VR treatment in patients with chronic phase. However, since it is not statistically significant, it will be necessary to conduct additional analysis on more research items in the future.

While the treatment duration of most of the included studies was short, there were many studies that increased the weekly treatment frequency. Nevertheless, the meta-regression analysis showed that the studies that increased frequency showed a smaller effect than the studies with lower treatment frequencies. In particular, there was a slight decrease in cases of more than four times. This demonstrates that chronic stroke patients require rest to learn movements. However, the number of studies included in this study was limited and the results were not statistically significant. Therefore, it is considered that there is a limit to interpretation, and it will be necessary to reanalyze more researches in future.

This study had several limitations. First, the lack of studies caused some difficulties performing a subgroup analysis. This is thought to be because we restricted the years of publication and only used three databases. For this reason, further meta-analysis will be required. Second, the type of VR program could also affect the therapeutic effect; however, the intervention types in the studies included in our analysis were mostly game programs, and there were limitations in categorizing these. Therefore, if more diverse training programs are developed in the future, it will be necessary to perform an analysis by program type. Third, even though VR training has been demonstrated to be effective at improving ADLs, because the number of studies included in the analysis was very small, there are limitations in generalizing the results. There have been very few researchers who have measured ADLs, and therefore, in the future, we recommend that researchers plan to study VR by investigating the effects of VR on ADLs.

## 5. Conclusions

This was a systematic review and meta-analysis to examine whether VR rehabilitation training helps to improve function in chronic stroke patients, and the results showed a moderate-sized effect. Moreover, VR rehabilitation training showed a similar effect for improving lower limb function as it did for upper limb function. Finally, we verified that VR training requires a duration of at least 8 weeks, and that occasional treatment is actually more effective than treatment every day.

This study has a moderate evidence to support the effect of VR on lower extremity function in patients with chronic stroke. Therefore, VR training would be helpful in improving functional outcomes with chronic stroke patients such as gait (speed, cadence, 10MWT, 6MWT), balance (BBS, TUG, postural sway), lower limb movement (FMA, RMI), lower limb strength, and lower limb muscle tone. However, the details on how to use VR program must be set according to the therapeutic goals.

## Figures and Tables

**Figure 1:** Study flow diagram of systematic review.

**Figure 2:** Funnel plot for publication bias.

**Figure 3:** Effect size of Virtual Reality-Based Rehabilitation Program.

**Figure 4:** Results of the meta-regression analysis by intervention duration (weeks).

**Figure 5:** Results of the meta-regression analysis by weekly intervention frequency.

**Table 1:** Strategy for electronic databases survey.

Electronic databases	Key words (DECS/MeSH)
EMBASE	('cerebrovascular':ab OR 'stroke':ab) AND 'virtual reality':ab = 632
OVID	((stroke or cerebrovascular) and virtual reality).ab. = 528
PubMed	(stroke[Title/Abstract] OR cerebrovascular[Title/Abstract]) AND virtual reality[Title/Abstract] = 507

**Table 2:** Methodological Quality of Trials (n = 21).

Study	score	1	2	3	4	5	6	7	8	9	10	11
Bang (2016)	4	0	1	0	1	0	0	0	0	0	1	1
Calabrò (2017)	9	1	1	1	1	0	1	1	1	1	1	1
Cho (2012)	5	1	1	0	1	0	0	0	1	0	1	1
Cho (2014)	7	0	1	1	1	0	0	1	1	0	1	1
da Silva Ribeiro (2015)	7	0	1	1	1	0	0	1	1	0	1	1
Fluet (2015)	4	1	0	0	1	0	0	0	0	1	1	1
In (2016)	8	1	1	1	1	0	0	1	1	1	1	1
Jang (2005)	5	0	1	0	1	0	0	0	1	0	1	1
Kim (2015)	4	0	1	0	1	0	0	0	0	0	1	1
Kiper (2014)	5	1	1	0	1	0	0	0	1	0	1	1
Lee D (2014)	5	1	1	0	1	0	0	1	0	0	1	1
Lee (2015)	5	1	1	0	1	0	0	0	1	0	1	1
Lee (2016)	6	1	1	0	1	0	0	1	1	0	1	1
Llorens (2015)	8	1	1	1	1	0	0	1	1	1	1	1
Park (2016)	8	1	1	1	1	1	0	1	0	1	1	1
Park (2017)	6	1	1	1	1	0	0	1	0	0	1	1
Sin (2013)	6	1	1	0	1	0	0	1	1	0	1	1
Singh (2013)	9	1	1	1	1	1	0	1	1	1	1	1
Song (2015)	3	1	1	0	0	0	0	0	0	0	1	1
Viana (2014)	9	1	1	1	1	1	1	1	1	0	1	1
Yom (2015)	6	1	1	0	1	0	0	1	1	0	1	1

PEDro items: 1 Eligibility criteria; 2 Random allocation; 3 Concealed allocation; 4 Baseline Comparability; 5 Blind subjects; 6 Blind therapists; 7 Blind assessors; 8 Adequate follow-up; 9 Intention to treat analysis; 10 Between-group statistical comparisons; 11 Point estimates and variability.

**Table 3:** General Characteristics of Included Trials.

Study	Mean age E(C)	No. of patients analyzed E(C)	Months since onset E(C)	VR Intervention	Control Intervention	Outcome Measures
Bang (2016) [10]	62.2 (63.2)	20 (20)	30.4 (31.6)	Wii board balance system: yoga, muscular strength exercise, aerobic exercise, balancing exercise 40 min*∗*3 d/w*∗*8 wks	low-speed treadmills 40 min*∗*3 d/w*∗*8 wks	Lt/Rt WB Ant/post WB Affected side -stance phase -swing phase Cadence

Calabrò (2017) [11]	60.0 (63.0)	12 (12)	8.0 (8.0)	VR+RAGT (robotic assist gait training) 45min*∗*5d/w*∗*8	RAGT (robotic assist gait training) 45min*∗*5d/w*∗*8	RMI POMA MAS

Cho (2012) [12]	65.2 (63.1)	11 (11)	12.5 (12.6)	Nintendo Wii balance training (balance Bubble, ski slalom, ski jump, soccer heading, table tilting, penguin slide 30 min + Standard training (PT, OT) 30 min *∗*5 d/w*∗*6 wks	Standard training (PT, OT) 30 min *∗*5 d/w*∗*6 wks	PSV-apeo PSV-mleo PSV-apec PSV-mlec BBS / TUG

Cho (2014) [13]	65.7 (63.5)	15 (15)	13.8 (15.3)	Treadmill training based real-world video recording: 30 min*∗*3d/w, 6 wks + PT (NDT, PNF) 30 min, OT (U/E ADL) 30 min, FES 20min *∗*5d/w*∗*6wks	Treadmill walking training: 30 min*∗*3 d/w, 6 wks + PT (NDT, PNF) 30 min, OT (U/E ADL) 30 min, FES 20 min *∗*5 d/w*∗*6 wks	AP, ML-PSV PSVM BBS / TUG Gait speed Cadence SLSP,(%) GC DLSP,(%) GC Step length Stride length

da Silva Ribeiro (2015) [14]	53.7 (52,8)	15 (15)	42.1 (60.4)	Nintendo (tennis, hula hoop, soccer, boxing games) 60 min*∗*2 d/w*∗*8 wks	Conventional therapy(stretching, trunk and scapular mobilization, balance, UL diagonal movement, gripping, gait) 60 min*∗*2 d/w*∗*8 wks	FMA SF-36

Fluet (2015) [15]	X (X)	10 (11)	60.0 (87.0)	Robotic/virtually simulated, arm and finger rehabilitation activities: 180 min*∗*4 d/w*∗*2 wks	Repetitive task practice on arm and finger activities: 180 min*∗*4 d/w*∗*2 wks	WMFT FMA-UE RGT

In (2016) [16]	57.0 (54.0)	13 (12)	12.5 (13.6)	(VR reflection therapy 30min + Conventional therapy: patient-specific NDT, PT, OT, ST 30 min)*∗* 5 d/w*∗*4wks	(Placebo VR 30min*∗* 5d/w*∗*4wks 30min + Conventional therapy: patient-specific NDT, PT, OT, ST 30min)*∗*5d/w*∗*4wks	BBS / FRTTUG EO APS, MLS, TSEC APS, MLS, TS10mWV

Jang (2005) [17]	59.8 (54.4)	5 (5)	13.8 (13.4)	VR(reaching, lifting, and grasping motor skills game) 60min*∗*5d/w*∗* 4wks	No treatment	BBT MFT FMA-UE

Kim (2015) [18]	X (X)	10 (7)	>6	Community-based virtual reality scene exposure combined with treadmill training: 30 min*∗*3d/w*∗*4wks + Conventional PT (muscle strengthening, balance training, and indoor and outdoor gait training): 60 min*∗*5d/w*∗*4wks	Over ground walking, stair walking, slope walking, and unstable surface walking for 570 m 30 min*∗*3 d/w*∗*4 wks + Conventional PT(muscle strengthening, balance training, and indoor and outdoor gait training): 60 min*∗*5 d/w*∗*4 wks	PSPL AP PSPL ML PSPL total APSS

Kiper (2014) [19]	63.1 (65.5)	23 (21)	>12	Reinforced feedback in virtual environment: grasping and reaching movement 120 min*∗*5 d/w*∗*4 wks	Exercises of various movements in a horizontal or vertical plane 120 min*∗*5 d/w*∗*4 wks	FMA-UE FIM Movement -Time(sec) -Speed (cm/sec) -Peak (n)

Lee D (2014) [20]	58.3 (65.4)	12 (12)	9.3 (8.9)	VRRE (Asymmetric training on hand): 30 min*∗*5 d/w*∗* 4 wks + Standard rehabilitation training: gait, strengthening 60 min*∗*5 d/w*∗*4 wks + FES 25 m in*∗*5 d/w*∗*4 wks	Symmetric training on hand: 30min*∗*5d/w*∗* 4wks + Standard rehabilitation training: NDT(gait, strengthening): 60 min*∗*5 d/w*∗*4 wks + FES 25 min*∗∗*5 d/w*∗*4 wks	FMA-UE BBT Grip strength MAS-UE

Lee H (2015) [21]	45.9 (49.2)	12 (12)	>6	VR training(sitting posture, knee bend & other leg knee extend, tightrope walking, penguin teeter-totter seesaw, balance skiing, rolling marble board, balance Wii) 30 min*∗*3 d/w*∗*6 wks + General exercise 60 min*∗*5 d/w*∗*6 wks	Task-oriented training (sit to stand from different heights, task training in standing, balance training on an unstable surface, lifting a leg in place, kicking a ball, stair climbing and descending) 30 min*∗*3 d/w*∗*6 wks + General exercise 60 min*∗*5 d/w*∗*6 wks	EOWB COP ECWB COP EONB COP ECNB COP -Path length, -velocity FRT

Lee S (2016) [22]	69.2 (73.1)	10 (8)	16.2 (17.0)	Virtual reality-based bilateral upper extremity training 30min*∗*3d/w*∗*6wks + Conventional OT 30min*∗*5d/w*∗*6wks	Watching an irrelevant video in a VR environment with bilateral upper extremity training 30 min*∗*3 d/w*∗*6 wks + Conventional OT 30 min*∗*5 d/w*∗*6 wks	JHFT BBT GPT Strength -biceps, triceps grip strength palmar pinch lateral pinch tip pinch

Llorens (2015) [23]	58.3 (55.0)	10 (10)	13.6 (19.6)	(Audiovisual feedback while performing a stepping task 30 min+ Conventional therapy 30 min)*∗*5 d/w*∗*4 wks	Conventional therapy (static standing exercises in different positions, task-specific reaching exercises, stepping tasks, static and dynamic balance exercises, walking exercises under different conditions) 60 min*∗*5 d/w,*∗*4 wks	BBS POMA-balance POMA-gait 10-m walking

Park (2016 ) [24]	61.6 (62.0)	15 (15)	>6	Wii Sports & Resort: bowling, table tennis, and canoeing 30 min*∗* 5 d/w*∗*4 wks + mental practice 5 min*∗*5 d/w*∗*4 wks	Wii Sports and Sports Resort games: bowling, table tennis, and canoeing games 30 min*∗* 5 d/w*∗*4 wks	FMA-UE BBT MAL-QOM

Park (2017) [25]	62.0 (65.3)	10 (10)	10.8 (14.1)	Xbox Kinect (Boxing, Table tennis, Soccer, Golf, Ski, Football) 30 min+ Conventional PT 30 min *∗*5 d/w, 6 wks	Conventional PT(NDT, PNF) 30 min *∗*5 d/w*∗* 6 wks	FMA-LE BBS TUG 10MWT

Sin (2013) [26]	71.8 (75.6)	18 (17)	7.2 (8.5)	(Xbox Kinect sports and adventure 30 min + standard training 30 min)*∗*3/w*∗* 6 wks	standard training: 30 min*∗*3 d/w*∗* 6 wks	ROM-UE FMA-UE BBT

Singh (2013) [27]	65.4 (67.0)	15 (13)	40.5 (34.9)	(Nintendo Balance: Bubble, Xbox 360 Kinect: Rally Ball 30min + standard PT) 90 min*∗*2 d/w*∗*6 wks	Standard PT (self-stretching and strengthening exercises, coordination and balance exercises, functional exercises) 120 min*∗*2 d/w*∗*6 wks	BI OBS 6MWT 30sSTS TUG T10mWT

Song (2015) [28]	51.4 (50.1)	20 (20)	14.8 (14.3)	Xbox Kinect Sport, Sport Season 2, Adventure, and Kinect Gunstringer 30 min *∗*5 d/w*∗*8 wks	ergometer training 30 min *∗*5 d/w*∗*8 wks	Affected side WB Forward LOS Backward LOS TUG 10MWT

Viana (2014) [29]	56.0 (55.0)	10 (10)	31.9 (35.0)	VR exercises for the UL (Wii Sports resort, Wii Play Motion, Let's Tap) 60 min*∗*3 d/w*∗*5 wks + tDCS (primary motor cortex) 13 min*∗*3 d/w*∗*5 wks	VR exercises for the UL(Wii Sports resort, Wii Play Motion, Let's Tap) 60 min*∗*3 d/w*∗*5 wks + sham tDCS (primary motor cortex) 13 min*∗*3 d/w*∗*5 wks	FMA-UL WMFT-time WMFT-FAS MAS Grip strength SSQOL SSQOL -UL%

Yom (2015) [30]	64.6 (78.1)	10 (10)	11.1 (11.6)	Virtual reality-based ankle exercise (VRAE): exercising on the floor, balance board, cushion ball, standing on one foot. 30 min*∗*5 d/w*∗*6 wks + Conventional PT 60 min*∗*5 d/w*∗*6 wks	Watching an environmental documentary irrelevant to ankle exercise 30 min*∗*5 d/w*∗*6 wks + Conventional PT 60 min*∗*5 d/w*∗*6 wks	MAS Tardieu scale TUG Velocity Cadence Step length Stride length Stance time % Swing time % Double limb support

RMI (Rivermead mobility index), MAS (modified Ashworth scale), PSV-apeo (postural sway velocity-AP eye open), PSV-mlec (postural sway velocity-ML eye close), BBS (Berg Balance Scale), TUG (Timed up and go test), AP-PSV (anteroposterior postural sway velocity), ML-PSV (mediolateral postural sway velocity), PSVM (postural sway velocity moment), SLSP (single limb support period), GC (gait cycle), DLSP (double limb support period), FMA (Fugl Myer Assessment), SF-36 (Short Form 36 Health Survey), WMFT (Wolf Motor Function Test), RGT (Reach to Grasp Test), FRT (functional reach test), EO-APS (eyes open anterior-posterior sway distance), EO-MLS (eyes open medial-lateral sway distance), EO-TS (eyes open total sway distance), EC-APS (eyes closed anterior-posterior sway distance), EC-MLS (eyes closed medial-lateral sway distance), EC-TS (eyes closed total sway distance), 10-m WV (10-m walking velocity), 10-m WV (10-m walking velocity), BBT (Box and Block Test), MFT (manual function test), PSP L (postural sway path length), PSPL (postural sway path length), PSPL (postural sway path length), APSS (average postural sway speed), FIM (functional independence measure), ECWB COP (eyes-closed wide base), EONB COP (eyes-open narrow base), FRT (functional reach test), JHFT (Jebsen-Taylor hand function test), GPT (grooved pegboard test), MAL-QOM (motor activity log-quality of movement), BI (Barthel index), OBS (Overall balance score), 6MWT (six-minute walk test), 30-s STS (thirty-second sit to stand test), T10-m WT (timed ten-meter walk test), LOS (limit of stability), WMFT (wolf motor function test), WMFT-FAS (functional ability), SSQOL-UL (stroke specific quality of life-upper limb).

**Table 4:** Effect size of Virtual Reality Based Rehabilitation Program on function.

Function	K	ES	SE	p-value	95% CI
Upper Limb Function	53	0.431	0.054	0.001	0.424–0.537

Lower Limb Function	74	0.424	0.045	0.001	0.336–0.513

Overall Function	6	0.545	0.149	0.001	0.253–0.837

**Table 5:** Effect size of Virtual Reality Based Rehabilitation Program on outcomes.

Outcomes	K	ES	SE	p-value	95% CI
Muscle tone	5	0.755	0.196	0.001	0.372–1.139

Muscle strength	7	0.750	0.177	0.001	0.403–1.098

ADL	3	0.627	0.199	0.002	0.237–1.018

ROM	10	0.517	0.114	0.001	0.294–0.741

Gait	30	0.445	0.070	0.001	0.309–0.582

Function	23	0.388	0.085	0.001	0.222–0.554

Balance	40	0.364	0.061	0.001	0.244–0.484

Kinematics	12	0.274	0.109	0.012	0.060–0.488
